RETRACTED

# BRD7 Acts as a Tumor Suppressor Gene in Lung Adenocarcinoma

**DOI:** 10.1371/journal.pone.0156701

**Published:** 2016-08-31

**Authors:** Yushun Gao, Bing Wang, Shugeng Gao

**Affiliations:** Department of thoracic surgical oncology, cancer institute (hospital), Chinese academy of medical sciences, Peking union medical college, Beijing, 100021, China; H. Lee Moffitt Cancer Center & Research Institute, UNITED STATES

## Abstract

Lung cancer is one of the most malignant tumors and the leading cause of cancer-related deaths worldwide. Among lung cancers, 40% are diagnosed as adenocarcinoma. Bromodomain containing 7 (BRD7) is a member of bromodomain-containing protein family. It was proved to be downregulated in various cancers. However, the role of BRD7 in lung adenocarcinoma is still unknown. Western blot and qRT-PCR was performed to measure the BRD7 expression in lung adenocarcinoma tissues and cells. CCK8 and migration assay was done to detect the functional role of BRD7 in lung adenocarcinoma. In this study, we showed that the expression of BRD7 was downregulated in lung adenocarcinoma tissues and cells. The lower of BRD7 levels in patients with lung adenocarcinoma was associated with shortened disease-free survival. Furthermore, overexpression of BRD7 inhibited lung adenocarcinoma cell proliferation and migration. Inhibition of BRD7 expression promoted cell proliferation and migration by activating ERK phosphorylation. Overexpression of BRD7 inhibited cyclin D and myc expression. Our findings are consistent with a tumor suppressor role for BRD7 in lung adenocarcinoma tumorigenesis.

## Introduction

Lung cancer, one of the most malignant tumors, was the leading cause of cancer-related deaths worldwide, with about 226,000 new cases in 2012 in the United States[1–5]. Among lung cancers, 40% are diagnosed as adenocarcinoma and the 5-year survival rate for lung adenocarcinoma patients is only 5–20% at later stages[6–9]. Despite recent advances in the molecular mechanisms and surgical and chemotherapeutic interventions, the prognosis of lung adenocarcinoma has not improved significantly[10, 11] Therefore, it is an urgent to identify an efficient and novel predictive marker for lung adenocarcinoma.

Bromodomain containing 7 (BRD7), also known as NAG4, BP75 or CELTIX1, is a member of bromodomain-containing proteins family[12–14]. Recent studies demonstrated that BRD7 was mostly located in the nucleus and regulated chromatin remodeling[15–17]. More importantly, increasing evidences showed that BRD7 were downregulated in many cancers such as epithelial ovarian carcinoma, breast cancer, nasopharyngeal cancer and colorectal carcinoma [18–21]. For example, Hu et al. showed that BRD7 acted as a tumor suppressor in osteosarcoma, and knockdown of BRD7 increased colony formation, tumor growth and cell proliferation of osteosarcoma[22]. Park et al. demonstrated that overexpression of BRD7 inhibited ovarian cancer cells invasion, apoptosis and viability[18]. However, the role of BRD7 in lung adenocarcinoma is still unknown.

RETRACTED

In our study, we demonstrated that the expression of BRD7 was downregulated in lung adenocarcinoma tissues and cells. Moreover, lower of BRD7 levels in patients with lung adenocarcinoma was associated with shortened disease-free survival. Overexpression of BRD7 inhibited lung adenocarcinoma cell proliferation and migration. Our findings demonstrated that BRD7 played a tumor suppressor role in lung adenocarcinoma tumorigenesis.

## Materials and Methods

### Tissue specimens and cell lines and cell transfection

Thirty frozen tissues from lung adenocarcinoma patients were obtained in our hospital between 2010 and 2012. All tissues were immediately snapped frozen at -80°C. All protocols were approved by the Ethics Committee of the cancer institute(hospital). Written informed consent from each patient was collected. Human lung adenocarcinoma cell lines (H1299, H23, SPC-A1 and A549) were obtained from the Cell Resource Center of Institute of Chinese Academy of Medical Sciences (Beijing, China), and keep in RPMI 1640 medium. BRD7 plasmid or mock vector was transfected by using Lipofectamine 2000 (Invitrogen, Carlsbad, CA) following to the manufacturer’s instruction.

### Cell proliferation and migration assay

CCK8 (Dojindo; Kumamoto, Japan) was performed to measure cell proliferation. Cells were cultured in 10% CCK-8 diluted in normal medium until visual color conversion occurred. Proliferation rates were detected at 0, 24 and 48 hours after transfection. For migration assay, a wound-healing assay was performed. An artificial wound was performed by using a 200-ll pipette tip. To measure migrated cells, pictures were taken at 0, 24 and 48 h.

### Western blot

Western blot was performed using standard methods. Protein samples were loaded on 12% SDS gels and then transferred to membranes (Millipore, Danvers, MA, USA). After blocked with 5% nonfat milk, membranes were incubated for 2 hours with the following antibodies: BRD7 and GAPDH (Abcam, Cambridge, MA, USA). Proteins were measured using the enhanced chemiluminescence system (GE Healthcare).

### RNA extraction and qRT-PCR

Total RNA was extracted from the tissues and cells using Trizol reagent (Invitrogen, Calsbad, CA, USA). qRT-PCR was performed to detect the BRD7 expression following previous methods on the iQ5 Real-Time PCR Detection System (Bio-Rad, California, USA). The sequences of the specific primers are shown: BRD7 sense: CTGGAGATGCCGAAGCACAC, anti-sense:TGGGATCCACAGGATGGAGA; GAPDH sense: AGCCACATCGCTCAGACAC, anti-sense: GCCCAATACGACCAAATCC.

RETRACTED

### Statistical analysis

Statistics was done by one-way ANOVA for comparing continuous variables of more than two groups, respectively. The data were shown as the mean±SD (standard deviation). P≤0.05 were regarded as being statistically significant.

## Result

### The expression level of BRD7 was downregulated in lung adenocarcinoma cell lines

The protein expression of BRD7 was downregulated in lung adenocarcinoma cell lines and lung adenocarcinoma tissue compared to the adjacent no-tumor tissue (Fig 1A and 1B). Meanwhile, the mRNA expression of BRD7 was also lower in four lung adenocarcinoma cell lines and one lung adenocarcinoma tissues compared to one adjacent no-tumor tissues (Fig 1C).

**Fig 1:** The expression level of BRD7 was downregulated in lung adenocarcinoma cell lines. (A) The protein expression level of BRD7 in four lung adenocarcinoma cell lines (H1299, H23, SPC-A1 and A549) and one lung adenocarcinoma tissues and adjacent no-tumor tissue was measured by Western blot. (B) The signal in each lane was quantified using ImageJ software and the ratio of BRD7 to GAPDH was determined. (C)The mRNA expression level of BRD7 in four lung adenocarcinoma cell lines (H1299, H23, SPC-A1 and A549) and one lung adenocarcinoma tissues and adjacent no-tumor tissue was measured by qRT-PCR.

### The expression level of BRD7 was downregulated in lung adenocarcinoma tissues

The mRNA expression of BRD7 was lower in lung adenocarcinoma tissues compared to adjacent no-tumor tissues (Fig 2A). The expression of BRD7 was downregulated in 22 cases (22/30, 73%) in comparison with the adjacent tissues (Fig 2B). Furthermore, tissues from lymph node metastases expressed lower levels of BRD7 compared to primary lung adenocarcinoma tissues and the adjacent normal tissue (Fig 2C). When correlated to disease outcome, lower of BRD7 levels in patients with lung adenocarcinoma was associated with shortened disease-free survival (hazards ratio = 0.36, Fig 3A). The protein level of BRD7 was also downregulated in lung adenocarcinoma tissues compared to adjacent no-tumor tissues (Fig 3B).

**Fig 2:** The expression level of BRD7 was downregulated in lung adenocarcinoma tissues. (A) Relative PBRD7 mRNA expression levels inlung adenocarcinoma tissues and their corresponding adjacent normal tissues. (B) qRT-PCR analysis of BRD7 expression in 30 pair’s lung adenocarcinoma tissues and their corresponding adjacent normal tissues. (C) Tissues from lymph node metastases expressed lower levels of BRD7 compared to primary lung adenocarcinoma tissues and the adjacent normal tissue.

RETRACTED

**Fig 3:** The protein expression level of BRD7 was downregulated in lung adenocarcinoma tissues. (A) Lower of BRD7 levels in patients with lung adenocarcinoma was associated with shortened disease-free survival (hazards ratio = 0.36). (B) The protein expression level of BRD7 was measured in lung adenocarcinoma tissues and their corresponding adjacent normal tissues using Western blot.

### Overexpression of BRD7 inhibited lung adenocarcinoma cell proliferation and migration

Western blot and real-time PCR analysis showed that BRD7 vector promoted the expression of BRD7 (Fig 4A and 4B). Overexpression of BRD7 inhibited lung adenocarcinoma cell line A549 proliferation and migration (Fig 4C, 4D and 4E).

**Fig 4:** Overexpression of BRD7 inhibited lung adenocarcinoma cell proliferation and migration. (A) The protein expression level of BRD7 was measured by using Western blot. (B) The mRNA expression level of BRD7 was measured by using qRT-PCR. (C) Overexpression of BRD7 inhibited lung adenocarcinoma cell line A549 proliferation. (D) Overexpression of BRD7 inhibited lung adenocarcinoma cell line A549 migration. (E) Relative ratio of wound closure per field is shown. *p<0.05 and ***p<0.001.

### Inhibition of BRD7 promoted ERK phosphorylation in lung adenocarcinoma

Western blot and real-time PCR analysis showed that BRD7 siRNA inhibited the expression of BRD7 (Fig 5A and 5B). Inhibition of BRD7 promoted the ERK phosphorylation in the A549 cells (Fig 5C). Knockdown of BRD7 expression increased the A549 cells proliferation, which could be blocked by U0126 (a MEK inhibitor) (Fig 5D). Knockdown of BRD7 expression increased the A549 cells migration, which could be blocked by U0126 (Fig 5E).

**Fig 5:** Inhibition of BRD7 promoted ERK phosphorylation in lung adenocarcinoma. (A) The protein expression level of BRD7 was measured by using Western blot. (B) The mRNA expression level of BRD7 was measured by using qRT-PCR. (C) Inhibition of BRD7 promoted the ERK phosphorylation in the A549 cells. (D) CCK8 analysis was used to measure the A549 cell proliferation. (E) Overexpression of BRD7 suppressed the ERK phosphorylation in the A549 cells. (F) Wound-healing assay was performed to measure the A549 cell migration. (G) Relative ratio of wound closure per field is shown. *p<0.05 and ***p<0.001.

### Overexpression of BRD7 inhibited Cyclin D and Myc expression

qRT-PCR analysis demonstrated that overexpression of BRD7 suppressed the cyclin D expressionin the A549 cells (Fig 6A). BRD7 overexpression inhibited the myc expression in the A549 cells. Moreover, knockdown of BRD7 expression increased cyclin D expression in the A549 cells, which could be blocked by U0126 (Fig 6C). In addition, knockdown of BRD7 expression increased myc expression in the A549 cells, which could be blocked by U0126 (Fig 6D).

RETRACTED

**Fig 6:** Overexpression of BRD7 inhibited Cyclin D and Myc expression. (A) Overexpression of BRD7 suppressed the Cyclin D mRNA expression in the A549 cells. (B) Overexpression of BRD7 suppressed the Myc mRNA expression in the A549 cells. (C) The mRNA expression level of Cyclin D was measured by using qRT-PCR in the A549 cells. (D) The mRNA expression level of Myc was measured by using qRT-PCR in the A549 cells.

## Discussion

As one of the most common cancers, lung adenocarcinoma was the leading cause of cancer death in the recent years. The most important prognostic factor for lung adenocarcinoma is the clinical stages[23, 24]. Unfortunately, even at the same clinical pathological stage, outcomes of patients vary considerably[25, 26]. This phenomenon is frequently observed in lung adenocarcinoma patients with clinical stage III and IV[27, 28]. Thereby, improving prognostic markers for clinical use is urgently needed.

In our study, we demonstrated that the expression of BRD7 was downregulated in lung adenocarcinoma tissues and cells. Moreover, the lower of BRD7 levels in patients with lung adenocarcinoma was associated with shortened disease-free survival. BRD7 was also downregulated in lung adenocarcinoma tissues compared to adjacent no-tumor tissues. Furthermore, overexpression of BRD7 inhibited lung adenocarcinoma cell proliferation and migration while inhibition of BRD7 expression promoted cell proliferation and migration by activating ERK phosphorylation. Overexpression of BRD7 inhibited cyclin D and myc expression. Our findings demonstrated that BRD7 played a tumor suppressor role in lung adenocarcinoma tumorigenesis.

BRD7 is a member of the bromodomain family and is encoded in a locus on chromosome 16q12[16, 29–31]. Recent studies have demonstrated that BRD7 acts as a tumor suppressor role in various cancers such as breast cancer, nasopharyngeal carcinoma, prostate cancer and osteosarcoma[19, 20, 22, 32]. For example, Hu et al showed BRD7 was downregulated in osteosarcoma, and knockdown of BRD7 increased colony formation, tumor growth and cell proliferation of osteosarcoma.[22]. BRD7 expression was correlated with patients’ survival time in osteosarcoma tissue. Park et al. demonstrated that overexpression of BRD7 inhibited ovarian cancer cells invasion, apoptosis and viability[18]. Drost et al. showed that BRD7 inhibited tumorigenicity by acting as a p53 cofactor in breast cancer [29]. However, the expression of BRD7 in lung adenocarcinoma is still unknown. In our study, the protein and mRNA expression of BRD7 was downregulated in four lung adenocarcinoma cell lines (H1299, H23, SPC-A1 and A549) and one lung adenocarcinoma tissues compared to one adjacent no-tumor tissues. Tissues from lymph node metastases expressed lower levels of BRD7 compared to primary lung adenocarcinoma tissues and the adjacent normal tissue. When correlated to disease outcome, lower of BRD7 levels was associated with shortened disease-free survival in patients with lung adenocarcinoma.

RETRACTED

We next studied the functional role of BRD7 in lung adenocarcinoma. BRD7 overexpression repressed lung adenocarcinoma cell proliferation and migration while knockdown of BRD7 expression promoted cell proliferation and migration. Previous study showed that BRD7 inhibited G1–S progression by transcriptionally regulating important molecules involved in ras/MEK/ERK and Rb/E2F pathways[33]. In this study, we also showed that inhibition of BRD7 could promote the ERK phosphorylation in the A549 cells. Moreover, knockdown of BRD7 expression increased the A549 cells proliferation and invasion, which could be blocked by U0126, a MEK inhibitor. These results demonstrated that downregulation of BRD7 promoted lung adenocarcinoma proliferation and migration through induction of ERK phosphorylation in the lung adenocarcinoma.

In conclusion, our results gave important clues for the functions of BRD7, indicating that BRD7 may present a promising candidate tumor suppressor gene in lung adenocarcinoma. Although the exact mechanism of BRD7 remains to be known, BRD7 may act as a potent target for therapeutic strategies for patients with lung adenocarcinoma.
